# Hsa_circ_0005379 regulates malignant behavior of oral squamous cell carcinoma through the EGFR pathway

This article has been retracted.

**DOI:** 10.1186/s12885-019-5593-5

**Published:** 2019-04-29

**Authors:** Wen Su, Yufan Wang, Feng Wang, Shuai Sun, Minghua Li, Yuehong Shen, Hongyu Yang

**Affiliations:** 1 Department of Oral and Maxillofacial Surgery, Peking University Shenzhen Hospital, No. 1120 Lianhua Road, Shenzhen, 518001 Guangdong China; 2 Peking University Shenzhen Hospital Clinical College, Anhui Medical University, Hefei, Anhui China; 3 Central laboratory, Peking University Shenzhen Hospital, Shenzhen, Guangdong China

**Keywords:** Oral squamous cell carcinoma, Circular RNAs, EGFR pathway, Cetuximab, Epithelial–mesenchymal transition

## Abstract

**Background:**

Oral squamous cell carcinoma (OSCC) is an oral and maxillofacial malignancy with a high incidence worldwide. Accumulating evidence indicates that circular RNAs (circRNAs) play a vital role in modulating tumor development. However, the mechanism of circRNA action in human OSCC remains largely unknown.

**Methods:**

By using high-throughput transcriptome sequencing technology, we conducted a comprehensive study of circRNAs in human OSCC. The effect of circRNA hsa_circ_0005379 on OSCC tissues and cell lines was monitored by qRT-PCR, Transwell assay, flow cytometry, and western blot analysis. Xenograft mouse models were used to assess tumor growth and animal survival.

**Results:**

We found that circRNA hsa_circ_0005379 expression is significantly lower in OSCC tissue compared to paired non-cancerous matched tissue and is associated with tumor size and differentiation. Overexpression of hsa_circ_0005379 effectively inhibits migration, invasion, and proliferation of OSCC cells in vitro and suppresses OSCC growth in nude mice in vivo. Mechanistic studies revealed that hsa_circ_0005379 may be involved in the regulation of the epidermal growth factor receptor (EGFR) pathway. Furthermore, we found that high expression of hsa_circ_0005379 could significantly enhance the sensitivity of OSCC to the cetuximab drug.

**Conclusions:**

Our findings provide evidence that hsa_circ_0005379 regulates OSCC malignancy and may be a new therapeutic target for OSCC treatment.

**Electronic supplementary material:**

The online version of this article (10.1186/s12885-019-5593-5) contains supplementary material, which is available to authorized users.

## Background

Oral squamous cell carcinoma (OSCC) is an invasive malignant tumor with different degrees of differentiation. The poor-differentiated OSCC has a tendency to metastasize to early lymph nodes [1]. It accounts for about 3% of the world’s malignant tumors [2]. Every year, 1.6 million people are diagnosed and 333,000 people die from head and neck squamous cell carcinoma (HNSCC), of which half the cases are OSCC [3]. Moreover, incidence rates of OSCC in developing countries are higher than developed countries [2]. The latest academic statistics shows that the five-year survival rate of patients with OSCC is about 60% [4], while the 5-year survival rate of patients with advanced cancer is even lower. OSCC has become a progressively serious global problem.

Circular RNAs (circRNAs) are a class of noncoding RNA molecules that do not have a 5′-end cap or 3′-end poly (A) tail. Previous reports have shown that circular RNAs are endogenous, stable, abundant, and conserved RNA molecules that can have cell type- or developmental stage-specific expression patterns in eukaryotic cells [5–7]. Studies have revealed the presence of differentially expressed circular RNA in various tumor tissues, which are significantly associated with distant metastases, TNM staging, and other clinical features [8, 9]. Including colon, gastric, and esophageal cancers [10, 11]. Studying features of circRNAs can provide new insights into tumor pathogenesis. However, literature on the expression of circular RNA in oral squamous cell carcinoma is limited.

To investigate the regulatory role of circRNAs in OSCC, high-throughput sequencing was used to screen differentially expressed circular RNA in paired OSCC tissues and adjacent normal tissue samples [12]. We found that hsa_circ_0005379 is an OSCC tumor suppressor gene associated with tumor size and differentiation. Upregalation of hsa_circ_0005379 effectively inhibits migration, invasion, proliferation of OSCC cells and angiogenesis formation in vitro, and suppresses OSCC growth in nude mice in vivo. We also found that hsa_circ_0005379 may be involved in the regulation of the epidermal growth factor receptor (EGFR) pathway by affecting EGFR expression. Moreover, our study showed that high expression of hsa_circ_0005379 combined with cetuximab can significantly promote OSCC cell apoptosis. Taken together, our findings provide evidence that hsa_circ_0005379 regulates cancer and may be a new therapeutic target for OSCC treatment.

## Methods

### Patients and tissue samples

All patient tissue samples were obtained from the Stomatological Center of Peking University Shenzhen Hospital (Shenzhen, China), between 2016 and 2018. Patients enrolled in the study was selected to rule out systemic disease and preoperative radiotherapy or chemotherapy. The histopathological grading of tumors was performed according to the 2018 World Health Organization classification criteria for head and neck cancer. The circular RNA profiling was obtained through high-throughput sequencing of four pairs of specimens. (Guangzhou Gene Denovo Biotechnology Co. Ltd., Guangzhou, China). This study was approved by the Ethics Committee of Peking University Health Science Center (IRB00001053–08043).

### Cell culture and transfection

Human OSCC cell lines SCC9, SCC15, SCC25, and CAL27 are gifts given by Wuhan University (Wuhan, China). Human oral keratinocyte (HOK) cells were obtained from the cell bank of the Chinese Academy of Sciences (Shanghai, China). All cells were cultured in Dulbecco’s modified Eagle medium (DMEM; Gibco, New York, USA). Human umbilical vein endothelial cells (HUVEC) and culture medium were bought from Procell Life Science and Technology Company (WuHan, China). All cell lines were cultured at 37 °C incubator with 5% CO_2_. The siRNAs for hsa_circ_0005379 were synthesized by RiboBio Co. Ltd. (Guangzhou, China). The siRNA sequences are as follows:

siRNA-1: 5′-CAAGGAAUGUAUCCUGUCA-3′;

siRNA-2: 5′-AAGGAUUUGCAAGGAAUGUAU-3′;

siRNA-3: 5′-GAUUUGCAAGGAAUGUAUCCU-3′.

Lipofectamine 3000 (Gibco, New York, USA) was used for siRNA transfection. All three siRNAs gave identical results.

### Lentivirus infection and monoclonal cell screening

The lentiviral plasmid containing GFP and puromycin-resistant gene was constructed by HanBio Co. Ltd. (Shanghai, China). Polybrene/medium mixture with packaged lentivirus was incubated with SCC25 and CAL27 cells for 48 h. After infection, the transduced cells were screened by puromycin (SCC25, 6 μg/ml; CAL27, 10 μg/ml; Qcbio Science & Technologies Co. Ltd. Shanghai, China). The screened cells were diluted and plated into 96-well plates to get a single cell per well. Monoclonal cells were verified by qRT-PCR. Fluorescence microscopy was used to observe the expression of GFP in infected cells.

### RNA preparation and qRT-PCR

Total RNA was extracted with an RNeasy Mini Kit (QIAGEN, Hilden, Germany). RNA was incubated with 3 U/mg RNase R (Epicenter) for 15 min at 37 °C. For reverse transcription, 500 ng of RNase R-treated RNA was reverse transcribed using Prime Script RT Master Mix (Takara Bio Inc., Kusatsu, Japan). PCR reactions were performed using PCR Master Mix (2×) (Thermo Fisher Scientific, Waltham, MA, USA). Primers used for qRT-PCR are listed as follows:

hsa_circ_0005379-F1: GCCCATACCTTTATCCACTC

hsa_circ_0005379-R1: GTCAACATTCCAGTCTCTTCCT

hsa_circ_0005379-F2: CCTAAGAAGACCACAATGCG

hsa_circ_0005379-R2:CCTCCGTAGTAAGGGTTTCG

β-actin-F: AAACTGGAACGGTGAAGGTG

β-actin-R: AGTGGGGTGGCTTTTAGGAT.

#### CCK-8 assay

Tumor cells were seeded into 96-well plates at 2 × 10^3^ cells per well. CCK-8 (Beyotime, Shanghai, China) was added at 10 μl/well at different time points and incubated for 1 h. The OD value at 450 nm absorbance was measured. To treat the cells with EGFR drugs, NSC228155 was added at the concentration of 29 μg/ml and incubated for 15 min. Cetuximab was added at the concentration of 10 μg/ml and incubated for 72 h.

### 5-ethynyl-2′-deoxyuridine (EdU) incorporation assay

Tumor cells were seeded at 4 × 10^3^ cells/well into 96-well plates and grown to logarithmic phase. Then EdU dye, PBS buffer, Apollo and Hoechst 33342 (Beyotime Biotechnology, Shanghai, China) were used to stain the cells, respectively. Images were taken randomly under a fluorescence microscopy. The cells were counted using Image J software.

### Co-cultivation experiment

The two types of OSCC cells conventionally stably transduced (tumor cells with high expression of hsa_circ_0005379) were cultured in 6-well plates in serum-free medium for 24 h. Supernatant medium was collected as conditioned medium. After trypsin digestion, HUVEC cells were centrifuged and the cells were resuspended in serum-free DMEM medium and counted. Then, 3 × 10 ^4^ cells were added to each well and the medium was adjusted to 100 μl using serum-free medium. In the lower chamber, two kinds of conditioned medium or two kinds of stably transduced cells cultured with serum-free DMEM medium were added. After 24 h, the medium was discarded and the cells were fixed in 4% paraformaldehyde and stained with crystal violet staining solution. The cells above the membrane were observed and photographed on an inverted microscopy.

### Tube formation assay

Matrigel was added to 24-well plates at a concentration of 200 μl/well and placed in an incubator for 1 h to solidify. The HUVECs were inoculated into the above 24-well plate, and the confluency is about 60% when the cells attached. The cells were cultured for 12 h by adding the above mentioned conditioned medium or OSCC cells overexpressing hsa_circ_0005379. The photographs were taken on an inverted microscopy.

### Flow cytometry

Annexin V-FITC Apoptosis Assay Kit (Beyotime Biotechnology Co. Ltd., Shanghai, China) was used to measure the cell apoptosis rate. Tumor cells were seeded into 6-well plates and grown to logarithmic phase. The cells were harvest by digestion and resuspended in 100 μl of 1 × annexin-binding buffer. 5 μl of annexin V and 1 μl of propidium iodide (PI) reagent were added to each well and incubated for 15 min. After incubation, 400 μl of 1 × annexin-binding buffer was added to stop staining. The apoptosis rate was finally measured using FACSCalibur flow cytometer (BD Biosciences, New York, USA).

### Hoechst 33258 staining experiment

Tumor cells were seeded at 4 × 10^5^ cells/well into 24-well plates and grown to logarithmic phase. Cells were then fixed using 4% paraformaldehyde and stained by Hoechst 33258 (Beyotime Biotechnology Co. Ltd., Shanghai, China). The morphology and staining of tumor cells nuclei were observed under an inverted fluorescence microscopy.

### Wound-healing assay

Cells were seeded in 6-well plates and cultured until confluent. Use a sterile 200 μl pipette to scratch the bottom of the 6-well plate. The exfoliated tumor cells were washed with PBS, and cell migration photographs were taken under a microscope at 0 h and 48 h, respectively.

### Migration and invasion assays

Migration and invasion experiments were performed using a Transwell chamber with or without Matrigel (Corning Life Sciences, NY, USA). The upper chamber is serum-free DMEM, and the lower chamber is DMEM containing 10% FBS. After 24 and 48 h of culture, tumor cells which passed through the chamber were fixed and stained by 4% paraformaldehyde and 0.1% crystal violet. Images were taken under an inverted microscopy.

### Western blot analysis

Cellular extracts were prepared at 4 °C in RIPA buffer (Beyotime Biotechnology, Shanghai, China). Western blot analysis was performed using commercial primary antibodies against the following proteins: Bcl-2 (1:2000; ab32124, Abcam), BAX (1:2000; ab32503, Abcam), MMP-9 (1:2000; ab38898, Abcam), cyclin D1 (1:2000; ab134175, Abcam), GAPDH (1:2000; ab8245, Abcam), vimentin (1:1000; 5741 T, CST), E-cadherin (1:1000; 3195 T, CST) N-cadherin (1:1000; 13,116 T, CST), β-catenin (1:1000; 8480 T, CST), EGFR (1:1000; 2085S, CST), CD31 (1:1000; 3528S, CST) and p-EGFR (1:1000; 3777S, CST). The bands were detected using HRP-conjugated secondary antibodies from Beyotime Biotechnology (Shanghai, China): goat anti-rabbit (1:1000, A0208) and goat anti-mouse (1:1000, A0216). Chemiluminescence was identified using Millipore chromogenic solution (MilliporeSigma, Burlington, MA, USA).

### Tumorigenesis and staining

Transduced CAL27 cells (2 × 10^7^ cells in 100 μl) were injected into 4-week-old Balb/c athymic nude mice (Siliake Jingda Experimental Animal Co. Ltd., Hunan, China).

The tumor volume of nude mice was measured and recorded according to V = πAB2/6 (V: tumor volume, A: the largest diameter, B: the perpendicular diameter). After 6 weeks, the nude mice were euthanized. Tumors of nude mice were dissected and tumor weights were measured. Tumor specimens were treated accordingly to perform hematoxylin and eosin (H&E) staining, Western blot, IHC staining.

### Image processing and statistical analysis

All images shown are wide-field microscopy images. Results in graphs are shown as the mean ± SEM from three independent experiments. All statistical data were analyzed using SPSS 17.0 software (SPSS, Chicago, IL, USA). Two-tailed Student’s *t*-tests were used to determine *P* values; *P* < 0.05 was considered significant.

## Results

### OSCC expresses low levels of hsa_circ_0005379

We determined the RNA levels of hsa_circ_0005379 by qRT-PCR and analyzed 37 pairs of clinical tissues. It is revealed that hsa_circ_0005379 expression was lower in cancerous tissues than adjacent normal tissues (Fig. 1a). We also investigated the expression level of hsa_circ_0005379 in four OSCC cell lines. We observed that hsa_circ_0005379 expression was remarkably downregulated in oral cancer cell lines compared to the expression in HOK cells (Fig. 1b). We also analyzed the correlation between clinicopathological features and hsa_circ_0005379 expression levels in 37 OSCC patients (Table 1). Results showed a negative correlation between OSCC tumor size (*P* = 0.0192) and differentiation grades (*P* = 0.0057). The ROC curve is shown in Fig. 1c.

**Fig. 1:** Hsa_circ_0005379 is downregulated in OSCC tissue specimens and cell lines. **a** The relative hsa_circ_0005379 expression level was determined in tissue specimens from patients with OSCC compared with adjacent normal tissues (*n* = 37) and (**b**) HOK, CAL27, SCC9, SCC15, and SCC25 cell lines by qRT-PCR. **c** ROC curve related to hsa_circ_0005379. Data are presented as mean ± S.E.M. of three independent experiments. Student’s *t-test*, *P < 0.05, ***P < 0.001

**Table 1:** Correlation between clinicopathological features and hsa_circ_0005379 expression levels in 37 OSCC patients

Parameter	No. of patients	Mean ± SEM	*P* value
Gender			
Male	27	9.7710 ± 0.4902	0.4225
Female	10	10.4700 ± 0.4649	
Age (yr)			
<60	13	10.9300 ± 0.6460	0.0741
≥ 60	24	11.9500 ± 0.2182	
Tumor size (cm)			
<5	30	11.4900 ± 0.3732	0.0192 *
≥ 5	7	9.2900 ± 0.9626	
Differentiation grade			
Well-moderate	12	11.8600 ± 0.5345	0.0057 **
Poor-undifferentiation	25	9.7540 ± 0.4225	
Lymph node status			
Negative	21	11.4000 ± 0.4521	0.5679
Positive	16	11.8200 ± 0.5790	
TNM stage			
I-II	13	10.4000 ± 0.6486	0.2432
III-IV	24	11.3000 ± 0.4333	

### Upregulation of hsa_circ_0005379 reduces proliferation and promotes apoptosis in OSCC cells

To investigate the role of hsa_circ_0005379 in regulating cell proliferation, we performed the CCK-8 assay on SCC25 and CAL27 cells overexpressing hsa_circ_0005379. After transducing SCC25 and CAL27 cells with hsa_circ_0005379 lentivirus, hsa_circ_0005379 expression levels increased approximately 4-fold and 6-fold, respectively (Additional file 1: Figure S1). The OD values were measured to determine the proliferation rate. The results revealed that with an increase in transduction time, hsa_circ_0005379 overexpressing cells showed a significant decrease in proliferation rate compared with control group (Fig. 2a). EdU staining was conducted to measure proliferation ratios to confirm these results. High expression of hsa_circ_0005379 in SCC25 and CAL27 decreased cell proliferation ratios by approximately 6 and 17% compared to the control group, respectively (Fig. 2b). Hoechst 33258 staining experiments showed that high expression of hsa_circ_0005379 also promoted apoptosis of tumor cells (Fig. 3).

**Fig. 2:** Upregulation of hsa_circ_0005379 inhibits OSCC cell proliferation. **a** SCC25 and CAL27 cells were transduced with mock control or lentivirus expressing hsa_circ_0005379. The CCK-8 assay was used to measure cell proliferation at different times after transduction. **b** The EdU incorporation assay was used to measure the proliferation ratio in control SCC25 and CAL27 cells and those overexpressing hsa_circ_0005379. Data are presented as means ± SEM of three independent experiments. Student’s *t*-test, *P < 0.05, **P < 0.01, ***P < 0.001. Scale bar, 20 μm

**Fig. 3:** Upregulation of hsa_circ_0005379 increases apoptosis rate of OSCC cells. Hoechst staining was performed on SCC25 and CAL27 cells transduced with mock control or lentivirus harboring hsa_circ_0005379. The proportion of apoptotic cells was quantified in SCC25 and CAL27 cells. Data are presented as means ± SEM of three independent experiments. Student’s *t*-test, ***P < 0.001. Scale bar, 20 μm

### Upregulation of hsa_circ_0005379 inhibits OSCC cell migration and invasion abilities

To determine the role of hsa_circ_0005379 in OSCC cell migration, wound healing assays were performed on control and hsa_circ_0005379 overexpression SCC25 and CAL27 cells. The scratch area at 0 and 48 h after wounding were measured and revealed that the wound-closure rate in hsa_circ_0005379 overexpression cells was significantly lower than control cells. Closure rate at 48 h in hsa_circ_0005379 overexpression cells was about 18% lower (SCC25; Fig. 4a) and 19.6% lower (CAL27; Fig. 4b) than those in the control cells. After 24 h of incubation, the number of cells that migrated to the lower chamber in a Transwell assay decreased from 850 to 600 and 300 in SCC25 and CAL27 cells overexpressing hsa_circ_0005379, respectively, (Fig. 4c). Taken together, these results suggest that OSCC cell migration ability was impaired by the upregulation of hsa_circ_0005379. To further study OSCC cell invasion ability, we also performed a Transwell invasion assay. After 48 h incubation, the number of cells across the chamber coated with Matrigel was measured. Overexpression of hsa_circ_0005379 strongly suppressed the invasiveness of SCC25 and CAL27 cells. In both cases, the invading hsa_circ_0005379 overexpression cells were about half the number of invading control cells (Fig. 4d). Co-culture experiments showed that the ability of tumor cells to induce HUVEC cell migration decreased after overexpressing hsa_circ_0005379 (Fig. 5a, b). Moreover, HUVEC tube formation assay was performed. Incubated with conditioned medium, overexpression of hsa_circ_0005379 resulted in less tubule formation (Fig. 5c). The experimental results showed that overexpression of hsa_circ_0005379 affects the ability of tumor cells to induce angiogenesis tube formation compared with the control group. These findings indicate that overexpression of hsa_circ_0005379 can not only inhibit migration and invasion of OSCC cells*,* but also influence the angiogenesis tube formation.

**Fig. 4:** Upregulation of hsa_circ_0005379 inhibits OSCC cell migration and invasion. **a**, **b** Wound healing assays were performed on (**a**) SCC25 and (**b**) CAL27 cells transduced with mock control or lentivirus expressing hsa_circ_0005379. The scratch area was measured at 0 and 48 h, and the percentage of closure at 48 h was calculated. **c**, **d** A Transwell assay was performed to quantify the migration and invasion ability of SCC25 and CAL27 cells transduced with mock control or lentivirus expressing hsa_circ_0005379. **c** Cells were seeded into the upper chamber (uncoated). After 24 h, those that crossed to the lower chamber were imaged and quantified. **d** Cells were seeded into the upper, Matrigel-coated chamber. After 48 h, cells that passed across the coated chamber were imaged and quantified. Data are presented as means ± SEM of three independent experiments. Student’s *t*-test, ***P < 0.001. Scale bar, 20 μm

**Fig. 5:** Upregulation of hsa_circ_0005379 attenuates the ability of OSCC cells to induce HUVEC cell migration and angiogenesis formation. **a**, **b** HUVEC cells were co-cultured with two kinds of conditioned medium (**a**) or SCC25 and CAL27 cells transduced with mock control or lentivirus expressing hsa_circ_0005379 (**b**). Data are presented as means ± SEM of three independent experiments. Student’s *t*-test, **P < 0.01, ***P < 0.001. Scale bar, 20 μm. **c** HUVEC cells were treated with or without conditioned medium for 12 h. Capillary-like tubes were visualized by phase contrast inverted microscopy and calculated

### Upregualtion of hsa_circ_0005379 enhances the sensitivity of OSCC to anticancer drug cetuximab

Since cetuximab is a commonly used anticancer drug for OSCC treatment, we performed a drug treatment experiment to investigate the effect of hsa_circ_0005379 on OSCC cell viability. Apoptosis rates in hsa_circ_0005379 overexpression cells were measured by annexin V-FITC/PI dual-label flow cytometry. We used flow cytometry to detect apoptosis in different treatment groups of SCC25 (Fig. 6a) and CAL27 (Fig. 6b). Early apoptotic rates in the mock group were 0.31 and 0.43% in SCC25 and CAL27 cells, respectively, while early apoptotic rates in the hsa_circ_0005379 group were 1.12 and 0.91% in SCC25 and CAL27 cells, respectively. Early apoptotic rates in the mock + cetuximab group were 17.88 and 15.22% in SCC25 and CAL27 cells, respectively, while early cell apoptotic rates in hsa_circ_0005379 + cetuximab group increased to 38.35 and 35.77% in SCC25 and CAL27 cells, respectively. Our experimental results show that high expression of hsa_circ_0005379 can promote the apoptosis of tumor cells. OSCC cells with high expression of hsa_circ_0005379 significantly increased the sensitivity of OSCC cells to cetuximab and promoted tumor cell apoptosis.

**Fig. 6:** Upregulation of hsa_circ_0005379 enhances the sensitivity of OSCC to anticancer drug cetuximab. **a**, **b** The SCC25 cells (**a**) and CAL27 cells (**b**) transduced with mock control or lentivirus expressing hsa_circ_0005379 were treated with or without cetuximab and analyzed by flow cytometry

### Hsa_circ_0005379 is involved in the regulation of the EGFR pathway

To explore the mechanism of hsa_circ_0005379 in regulating OSCC, we examined the expression level of related proteins. The Bcl-2 gene is an oncogene that has an inhibitory effect on apoptosis. BAX is an apoptosis-promoting protein in the BCL-2 family. Overexpression of BAX antagonizes the protective effect of BCL-2 and causes cell death [13–15]. MMP-9 is capable of degrading collagen, gelatin, fibronectin, laminin, and dissolving the basement membrane, thereby promoting migration and invasion of tumor cells [16]. The main function of cyclin D1 is to promote cell proliferation and gene transcription. Cyclin D1 promotes the cell cycle from the G1 phase to the S phase by binding to and activating the cyclin-dependent kinase CDK4, which is unique to the G1 phase. Cyclin D1 has been recognized as a proto-oncogene. The overexpression of Cyclin D1 is associated with malignant transformation [17]. Our results showed that overexpression of hsa_circ_0005379, BAX was upregulated, whereas Bcl-2, MMP-9, and cyclin D1 were downregulated (Fig. 7a). Epithelial–mesenchymal transition (EMT) refers to the biological process by which epithelial cells are transformed into mesenchymal phenotype cells by a specific procedure. Through EMT, epithelial cells lose cell polarity and epithelial phenotypes such as attachment to the basement membrane, and thus obtain higher interstitial phenotypes such as migration, invasion, anti-apoptosis, and ability to degrade extracellular matrix. EMT is an important biological process for the migration and invasion of epithelial-derived malignant cells [18]. Here, to evaluate the EMT process, we overexpressed hsa_circ_0005379 and detected EMT markers by western blot analysis. Compared to control OSCC cells, hsa_circ_0005379 overexpression cells showed decreased expression of vimentin and N-cadherin and increased expression of E-cadherin and β-catenin (Fig. 7b). Taken together, hsa_circ_0005379 participates in the EMT process and affects cell proliferation and invasion by regulating the expression levels of several key proteins.

**Fig. 7:** Up- or downregulation of hsa_circ_0005379 alters the expression levels of key proteins involved in cell proliferation, apoptosis, invasion, and the EGFR signaling pathway. **a**, **c** SCC25 and CAL27 cells were subjected to either overexpression (**a**) or knockdown (**c**) of hsa_circ_0005379 and cell extracts were immunoblotted with the indicated antibodies. **b** Key EMT protein levels were detected by western blotting after upregualtion of hsa_circ_0005379 in SCC25 and CAL27 cells. **d**, **e** EGFR and p-EGFR protein levels were detected by western blotting after down- (**d**) or upregulation (**e**) of hsa_circ_0005379. **f** The SCC25 and CAL27 cells were treated with EGFR inhibitor cetuximab or agonist NSC. The expression levels of hsa_circ_0005379 were quantified by qRT-PCR. Data are presented as means ± SEM of three independent experiments. Student’s *t*-test, n.s., not significant

Additionally, we used siRNA to knockdown hsa_circ_0005379 in SCC25 and CAL27 cells. The knockdown efficiency is about 70% in SCC25 and 85% in CAL27 (Additional file 1: Figure S2). The expression levels of BAX, Bcl-2 and MMP-9 are inversely correlated with hsa_circ_0005379 expression (Fig. 7c). Western blot results showed that EGFR and p-EGFR expression levels were increased after hsa_circ_0005379 knockdown (Fig. 7d), while EGFR and p-EGFR expression levels were decreased after hsa_circ_0005379 overexpression (Fig. 7e). These results suggest that manipulating expression levels of hsa_circ_0005379 will influence the EGFR pathway. We used EGFR pathway agonists (NSC228155) and inhibitors (cetuximab) at the indicated times and concentrations to alter the expression level of phosphorylated EGFR in the cells and then detected the corresponding hsa_circ_0005379 expression level by qRT-PCR. We found no significant change in hsa_circ_0005379 expression levels (Fig. 7f). Moreover, the proliferation differences between hsa_circ_0005379 overexpression and knockdown cell lines treated with EGFR inhibitor cetuximab or agonist NSC in different time points have been investigated, which is shown in Additional file 1: Figure S3. The above results indicate that hsa_circ_0005379 may be located upstream of the EGFR pathway and regulate the expression level of EGFR.

### Upregulation of hsa_circ_0005379 suppresses the growth of OSCC cells in vivo

To establish a xenograft tumor model, we injected CAL27 cell lines in nude mice. Tumors in the hsa_circ_0005379 overexpression group were considerably smaller than those in the empty-vector group (Mock, Fig. 8a). The tumor growth curve and final weight of the nude mice were suppressed in the hsa_circ_0005379 overexpression group relative to the control (Fig. 8b, c). Moreover, the H&E staining (Fig. 8d) and western blot (Fig. 8e) showed that the angiogenesis marker CD31, EGFR and p-EGFR were downregulated when hsa_circ_0005379 was overexpressed. Immunohistochemical (IHC) (Fig. 8f) staining of xenograft tumors showed that vimentin was downregulated in hsa_circ_0005379 overexpressing tumors, while E-cadherin was upregulated, which supported the western blot results. Expression of EGFR was downregulated in hsa_circ_0005379 overexpression tumors compared with the control group. Collectively, these results showed that hsa_circ_0005379 is crucial for tumor growth.

**Fig. 8:** Upregulation of hsa_circ_0005379 inhibits tumorigenesis. **a** Images of nude mice bearing xenograft tumors generated using CAL27 stable cells and of surgically removed tumors. **b** Tumor growth curve changes in tumor volume weeks after injection. **c** Tumor weight plots of mock and hsa_circ_0005379 overexpression groups. **d** H&E staining of xenograft tumors. **e** The expression levels of CD31, EGFR and p-EGFR in the experimental groups were determined by western blot. **f** Immunohistochemical (IHC) staining of xenograft tumors. Data are presented as means ± SEM of three independent experiments. Student’s *t*-test, **P < 0.01. Scale bars, 50 μm

## Discussion

OSCC is a common malignancy in the head and neck. About 540,000 new patients are diagnosed each year. Its high incidence rate poses a serious challenge to public health [19, 20]. Early and well-differentiated OSCCs usually achieve good results through active surgical treatment. However, for the advanced and poorly differentiated OSCC, even treated by surgical treatment, radiation therapy or chemotherapy, the five-year survival rate of the patients is only about 60% [21]. When the distant metastasis occurs, the patients’ survival and quality of life is even more difficult to guarantee [22].

CircRNAs is a very peculiar product in the process of the transmission and function of life genetic information. The current research shows that circRNA is also subject to the central law. Due to the particularity of the structure, circRNA has a unique function different from traditional linear nucleic acid molecules [23]. Functional circRNAs have been identified to act as microRNA sponges and RNA-binding protein (RBP) sequestering agents, as well as transcriptional regulators [24]. These multiple functional roles indicate great potential for circRNAs in biological applications. A growing number of studies have shown that circRNAs play a regulatory role in the tumor progression [9, 25–27].

Like other malignancies, the occurrence and development of OSCC is a series of complex biological cellular processes involved with coding and noncoding genes [28]. Recently, the regulatory role of circRNAs in OSCC has also begun to attract attention. Chen et al. found that circRNA_100290 can bind miR-29 through endogenous competition, thereby eliminating miR-29 inhibition of CDK6 and promoting the proliferation of OSCC cells [29]. Research on circRNAs in OSCC has just begun and further research in OSCC-specific circRNA expression is needed. In this study, high-throughput circRNA microarray technology was used to screen differentially expressed circRNA in four pairs of cancer tissues of OSCC patients. The series of cytological experiments confirmed that changing the expression level of hsa_circ_0005379 can affect the malignant biological behavior of OSCC cells. The western blot assay detected significant changes in proliferation and apoptosis. EMT plays an important role in the process of tumor invasion. We detected changes in E-Cadherin, β-Catenin, and other core indicators that are consistent with our invasion experiment results. The ability of angiogenesis is closely related to the occurrence and development of tumors. The stronger the angiogenic ability, the greater the possibility of tumor cell proliferation and distant metastasis. Our experiment found that after overexpressing hsa_circ_0005379, the ability of tumor cells to induce HUVECs to form blood vessels was significantly lower than that of the control group. Tumor angiogenesis can be evaluated from the levels of CD31, also known as platelet endothelial cell adhesion molecule-1 (PECAM-1/CD31). The richer the CD31 content, the faster the tumor proliferation rate. Our experimental results showed that after overexpression of hsa_circ_0005379, the CD31 content in nude mice was significantly lower than that in the control group, indicating that the differential expression of hsa_circ_0005379 affected the angiogenesis of tumor cells.

By knocking down hsa_circ_0005379 in SCC25 and CAL27 cell lines using siRNA, we found that the level of proliferation-related apoptosis protein were changed. However, the results of cytological experiments such as CCK-8, wound healing assay, and Transwell assays were not significantly different, probably due to the low level of hsa_circ_0005379 in OSCC lines and the inherent high degree of malignancy of SCC25 and CAL27 cells.

EGFR is a tyrosine kinase type I receptor whose family members include four homologous receptors: EGFR (HER1), HER2, HER3, and HER4. Studies have shown a high or abnormal expression of EGFR in many solid tumors, indicating that EGFR is involved in the malignant biological behavior of tumor cells [30, 31]. Upregulation of EGFR is closely related to early metastasis and poor prognosis. Over 90% of patients with head and neck squamous cell carcinoma test positive for EGFR [32]. In this experiment, the expression level of EGFR protein in OSCC cell lines SCC25 and CAL27 was significantly changed by overexpression or knockdown of hsa_circ_0005379, indicating that hsa_circ_0005379 can regulate the EGFR pathway. Using EGFR pathway agonists and inhibitors to alter the expression levels of phosphorylated EGFR in the cells, we found only weak expression changes of hsa_circ_0005379 that were not statistically significant. This indicates that hsa_circ_0005379 may be located upstream of the EGFR pathway and regulate EGFR expression levels. Based on the high expression of EGFR in OSCC, a series of targeted therapeutics for EGFR have been developed [33, 34].

Cetuximab is a recombinant human murine chimeric IgG1 monoclonal antibody, which has high affinity for EGFR, inhibits cell cycle progression, and induces tumor cell apoptosis by specifically binding to the extracellular EGFR domain. This reduces the production of MMPs and vascular endothelial growth factors, and inhibits tumor invasion and metastasis. Cetuximab has shown good clinical efficacy and tolerability for EGFR expression in head and neck cancers [35, 36]. This study found that changes in early apoptotic rates is not obvious in cells after high hsa_circ_0005379 expression in SCC25 and CAL27 cell lines. However, when cetuximab was added after overexpressing hsa_circ_0005379 in SCC25 and CAL27 cells, the early apoptotic rate of the cells significantly increased to 38.35 and 35.77%, respectively. This indicates that high hsa_circ_0005379 expression increases cetuximab sensitivity and provides a new potential target for OSCC anticancer drugs design in the future.

Using software, we also identified possible miRNA targets of hsa_circ_0005379, including hsa-miR-145, hsa-miR-182. However, the mechanisms still need to be investigated in subsequent experiments. To date, only a few functional circRNAs have been reported in OSCC. Therefore, more effort is needed to elucidate the functions and key mechanisms of OSCC-specific circRNAs, so that circRNAs can be used effectively in translational and precision medicine.

## Conclusions

Hsa_circ_0005379 is an OSCC tumor suppressor gene associated with tumor size and differentiation. Upregulation of hsa_circ_0005379 effectively inhibits migration, invasion, proliferation of OSCC cells and angiogenesis formation in vitro, and suppresses OSCC growth in nude mice. Moreover, hsa_circ_0005379 may be involved in the regulation of the EGFR pathway by affecting EGFR expression. Taken together, our findings provide evidence that hsa_circ_0005379 regulates malignant behavior of OSCC and may be a new therapeutic target for OSCC treatment.

## Additional file

Additional file 1: **Figure S1.** Description of data: Generation of SCC25 and CaL27 stable cell lines. **Figure S2.** The knockdown efficiency of siRNA against hsa_circ_0005379. **Figure S3.** Up- or downregulation of hsa_circ_0005379 affects cell proliferation. (PDF 7285 kb)
